The article "Beneficial Role of HO-1-SIRT1 Axis in Attenuating Angiotensin II-Induced Adipocyte Dysfunction" was retracted in 2021. Reasons: duplicate publication; concerns about the data.

# Beneficial Role of HO-1-SIRT1 Axis in Attenuating Angiotensin II-Induced Adipocyte Dysfunction

**DOI:** 10.3390/ijms20133205

**Published:** 2019-06-29

**Authors:** Hari Vishal Lakhani, Mishghan Zehra, Sneha S. Pillai, Nitin Puri, Joseph I. Shapiro, Nader G. Abraham, Komal Sodhi

**Affiliations:** 1 Department of Surgery, Internal Medicine, and Biomedical Sciences, Marshall University Joan C. Edwards School of Medicine, Huntington, WV 25701, USA; 2 Department of Pharmacology, New York Medical College, Valhalla, NY 10595, USA

**Keywords:** angiotensin II, mineralocorticoid receptor, heme oxygenase 1, sirtuin 1, adipocytes, oxidative stress

## Abstract

Background: Angiotensin II (Ang II), released by the renin–angiotensin–aldosterone system (RAAS), contributes to the modulatory role of the RAAS in adipose tissue dysfunction. Investigators have shown that inhibition of AngII improved adipose tissue function and insulin resistance in mice with metabolic syndrome. Heme Oxygenase-1 (HO-1), a potent antioxidant, has been demonstrated to improve oxidative stress and adipocyte phenotype. Molecular effects of high oxidative stress include suppression of sirtuin-1 (SIRT1), which is amenable to redox manipulations. The mechanisms involved, however, in these metabolic effects of the RAAS remain incompletely understood. Hypothesis: We hypothesize that AngII-induced oxidative stress has the potential to suppress adipocyte SIRT1 via down regulation of HO-1. This effect of AngII will, in turn, upregulate mineralocorticoid receptor (MR). The induction of HO-1 will rescue SIRT1, hence improving oxidative stress and adipocyte phenotype. Methods and Results: We examined the effect of AngII on lipid accumulation, oxidative stress, and inflammatory cytokines in mouse pre-adipocytes in the presence and absence of cobalt protoporphyrin (CoPP), HO-1 inducer, tin mesoporphyrin (SnMP), and HO-1 inhibitor. Our results show that treatment of mouse pre-adipocytes with AngII increased lipid accumulation, superoxide levels, inflammatory cytokine levels, interleukin-6 (IL-6) and tumor necrosis factor α (TNFα), and adiponectin levels. This effect was attenuated by HO-1 induction, which was further reversed by SnMP, suggesting HO-1 mediated improvement in adipocyte phenotype. AngII-treated pre-adipocytes also showed upregulated levels of MR and suppressed SIRT1 that was rescued by HO-1. Subsequent treatment with CoPP and SIRT1 siRNA in mouse pre-adipocytes increased lipid accumulation and fatty acid synthase (FAS) levels, suggesting that beneficial effects of HO-1 are mediated via SIRT1. Conclusion: Our study demonstrates for the first time that HO-1 has the ability to restore cellular redox, rescue SIRT1, and prevent AngII-induced impaired effects on adipocytes and the systemic metabolic profile.

## 1. Introduction

Classically, the RAAS has been described as a multi-organ endocrine axis that is governed by a negative feedback loop where elevated circulating AngII inhibits renal renin release. A large body of evidence, today, supports the notion that apart from regulating cardiac, vascular, and renal functions, the RAAS operates in nervous, immunological, and reproductive tissues [1]. Visceral adipose tissue (VAT), classified as an endocrine organ, is the latest to be shown to express and to be regulated by the RAAS [2]. VAT expresses all components of the RAAS, including angiotensinogen [3,4], renin [5], and aldosterone synthase (CYP11B2) [6]. Excess VAT underlies obesity, whose global burden is reflected in sheer numbers; 39% of the adult population is overweight, while 13% is obese [7]. Evidence suggests that RAAS blockade reduces obesity-related cardiovascular and renal complications, alleviates insulin resistance, and facilitates adipocyte differentiation [8,9,10,11]. AngII has been shown to reduce proliferation and increase lipid accumulation in mouse pre-adipocytes in culture. Recent studies have also shown that increased AngII in animals with Goldblatt’s hypertension is associated with increased visceral adiposity and reduced plasma adiponectin levels [9]. Aldosterone synthase (CYP11B2) and MR [12], which are critical RAAS components, also affect adipocyte structure and function [13]. MR blockade reduces adiposity-related cardiovascular and hepatic complications and has been shown to facilitate adipocyte differentiation [8,9,10,11]. MR-dependent adipogenesis has been demonstrated in mouse pre-adipocytes in response to aldosterone [14]. A direct effect of the RAAS on VAT/adipocyte structure and function, however, remains unresolved and the mechanisms involved in the RAAS function are not clearly understood.

Increased VAT mass promotes inflammatory infiltration with compromised secretion of protective adipokines, like adiponectin. Thus, VAT hypertrophy launches a complex patho-physiological maladaptive response characterized by a systemic spillover of inflammatory and oxidative mediators, reduced secretion of protective adipokines, and increased circulating levels of glucose. A cumulative line of evidence suggests that redox imbalance and chronic oxidative stress increase adipogenesis and precipitate adipocyte dysfunction [15]. The RAAS has been reported to increase lipid accumulation [16], an effect attributed to RAAS-induced redox imbalance. Molecular effects of high oxidative stress include suppression of SIRT1, which is amenable to redox manipulations [17]. Studies have shown that SIRT1 regulates adipogenesis in murine adipocytes. In the model of oxidative stress, SIRT1 over-expression and/or an exogenous antioxidant prevents redox-induced adipocyte hypertrophy and dysfunction [18]. To this end, studies from our lab have documented that upregulation of the endogenous heme­–heme oxygenase system (HO) reduces adipogenesis in murine pre-adipocytes and human mesenchymal stem cells [19,20,21]. Previous studies have documented the antioxidant properties of the HO system and HO-1 induction via CoPP reduces visceral adiposity and ablates metabolic imbalance in obese and diabetic mice [22,23,24,25,26].

Based on these observations, we propose to explore the mechanistic link between VAT-specific overactive RAAS and eventual development of adipocyte and metabolic dysfunction via increase in cellular oxidative stress. We hypothesize that AngII-induced oxidative stress has the potential to downregulate adipocyte SIRT1 via suppression of HO-1. We further hypothesize that HO-1 induction will provide an antioxidant setting, thus rescuing cellular SIRT1 and preventing adipocyte dysfunction. This study, for the first time, will demonstrate a negative regulatory effect of the HO-1-SIRT1 axis, which will improve the effects mediated by AngII on the adipocyte phenotype. Thus, the overall objective of this proposal is to uncover the molecular interplay between AngII, HO-1, and SIRT1 as it pertains to the regulation of adipocyte structure and function, eventually affecting the systemic metabolic homeostasis.

## 2. Results

### 2.1. Effects of HO-1 on AngII-Induced Alteration on Adipocyte Phenotype 

The dose-dependent effect of AngII demonstrated that 10 uM was the optimal concentration in increasing lipogenesis in 3T3-L1 cells, as previously published [9]. Our RT-PCR analysis showed significantly reduced expression of HO-1 in response to AngII treatment, as compared to the control group treated with adipogenic media alone (Figure 1A). As expected, treatment with CoPP induced increased expression of HO-1, as compared to AngII-treated murine adipocytes. Interestingly, the expression of HO-1 was increased by treatment with SnMP alone and CoPP and SnMP together. However, these findings are not surprising, as SnMP, which induced a significant increase in HO-1 expression, remains a potent inhibitor of HO activity, as shown previously [27,28,29]. Lipid accumulation, measured as the relative absorbance of Oil Red O staining in murine adipocytes, demonstrated that AngII-induced increased lipogenesis, as compared to the control group treated with adipogenic media alone and 3T3-L1 cells treated with SnMP alone (HO-inhibitor) (Figure 1B). SnMP treatment alone induced significant lipid accumulation as compared to the control treated with adipogenic media alone. This effect, induced by SnMP or AngII treatment alone, was significantly alleviated by the induction of the antioxidant HO-1 system using CoPP, an effect reversed by the treatment with SnMP (HO-inhibitor) (Figure 1B). Apart from that, mRNA expression of fatty acid synthase (FAS), a marker of lipid accumulation, was significantly upregulated in SnMP-treated cells, which was even further increased by AngII treatment, as compared to the control (Figure 1C). This increase was attenuated by CoPP, which was reversed by concomitant treatment with SnMP (Figure 1C). Furthermore, our results demonstrated that treatment with AngII significantly increased triglyceride levels as compared to the control, which was improved by HO-1 induction (Figure 1D). Concurrent exposure to the HO-1 inhibitor (SnMP) reversed the effect, observed by CoPP causing an increase in triglycerides levels, similar to AngII-induced triglyceride increase. We next evaluated the mRNA expression of the marker of mitochondrial biogenesis, PGC-1α, which showed significant downregulation by the treatment with SnMP alone and by AngII treatment, as compared to control with adipogenic media alone (Figure 1E). The expression was improved by the induction of CoPP, which was further reversed when treated concurrently with SnMP (Figure 1E). Apart from that, our results demonstrated a significant increase in the mRNA expression of inflammatory marker IL-6 by treatment with SnMP alone, which was further exacerbated by AngII treatment as compared to the control (Figure 1F). This increase was attenuated by CoPP, which was reversed by concomitant treatment with SnMP (Figure 1F).

### 2.2. Effect of AngII on Mechanistic Interplay between HO-1/SIRT1 Axis in Mouse Adipocyte with or without HO-1 Induction

Our next set of experiments examined the AngII-induced molecular disruptions involved in causing altered adipocyte phenotype. Our Western blot analysis showed that treatment with CoPP induced increased expression of HO-1, as compared to AngII-treated murine adipocytes (Figure 2A). Interestingly, the protein levels of HO-1 were also increased by the treatment with CoPP that also received the SnMP (Figure 2A). However, these findings are not surprising, as SnMP, which induced a significant increase in HO-1 expression, remains a potent inhibitor of HO activity, as shown previously [27,28,29]. We next examined the effect of AngII treatment on the expression of SIRT1 in 3T3-L1 cells. Our Western blot analysis demonstrated that the treatment with AngII induced significantly reduced expression of SIRT1 as compared to controls, which was rescued by the induction of HO-1 (Figure 2B). However, the improved expression of SIRT1 was consequently decreased by the treatment with SnMP. Aldosterone synthase (CYP11B2), a critical RAAS component causing upregulation of MR, also affected adipocyte phenotype [30]. Our results further demonstrated that treatment with AngII stimulated the expression of CYP11B2, an effect negated by treatment with CoPP (Figure 2C). The expression of CYP11B2 was further increased by treatment of murine adipocytes with CoPP that were also exposed to SnMP. Apart from that, our results showed increased expression of MR, induced by the treatment with AngII, as compared to the control (Figure 2D). This increase was significantly negated by treatment with CoPP, which was again reversed by subsequent treatment with SnMP. Our Western blot analysis further demonstrated that AngII also significantly reduced insulin receptor-β (IR-β) expression, which was significantly improved by treatment with CoPP (Figure 2E). IR-β expression was suppressed significantly by treatment with CoPP that also received the SnMP. In concordance with these findings, we also performed RT-PCR analyses for the mRNA expression of SIRT1, CYP11B2, and MR in our murine pre-adipocytes. The findings were similar to our results from our Western blot analysis, with an addition of the SnMP-alone-treated experimental group, which showed significant upregulation in the expression of CYP11B2 and MR and also a significant reduction in SIRT1 expression, as compared to the control (Figure S1A–C). Our results also showed significant upregulation in expression of angiotensin II receptor type 1 (AT1R) by treatment with SnMP alone and more so by AngII treatment, as compared to the control (Figure S1D). The treatment with CoPP demonstrated significantly lower AT1R expression, which was reversed by consequent treatment with SnMP.

### 2.3. Effect of AngII in CM Obtained from Mouse Adipocytes with or without HO-1 Induction

The incubation of murine adipocytes with dihydroethidium (DHE) to measure superoxide levels (indicator of ROS) significantly showed upregulated levels by SnMP alone and a further significant increase in the AngII-treated group, as compared to the control treated with adipogenic media only (Figure 3A). The treatment with CoPP alone demonstrated significantly lower superoxide levels, which was consequently reversed by treatment with SnMP, indicating that upregulation of HO-1 is required for reduction in this oxidative marker. We next examined the effect of AngII on inflammatory markers in murine adipocytes. Conditioned media (CM) obtained from the treated 3T3-L1 cells flasks, demonstrated that the levels of key inflammatory markers, IL-6 and TNF-α, were significantly increased with AngII treatment, as compared to control and SnMP treatment alone (Figure 3C,D). The levels of these inflammatory markers were attenuated by treatment with CoPP, implying that the attenuation was dependent on HO-1 induction. Conversely, the levels of these inflammatory markers were upregulated in the CM of the cells treated with CoPP and exposed to SnMP. Furthermore, adiponectin levels were reduced significantly in CM in response to treatment with SnMP alone, which was further significantly decreased by AngII, as compared to the control (Figure 3D). However, treatment with CoPP improved adiponectin levels, an effect reversed by subsequent treatment with SnMP. 

### 2.4. Effect of AngII with or without HO-1 Induction and SIRT1 Knockdown on Lipogenesis and FAS Levels in Mouse Adipocytes

To assess whether HO-1 requires the participation of SIRT1 to mediate and/or amplify its actions, we studied the effect of SIRT1 siRNA and SIRT plasmid in 3T3-L1 cells treated with AngII. Our results showed that AngII increased lipid accumulation, measured as the relative absorbance of Oil Red O staining in murine adipocytes, and expression of FAS; this effect of AngII treatment was significantly negated by treatment with CoPP (Figure 4A and Figure 4B, respectively). Interestingly, concurrent treatment with CoPP and SIRT1 siRNA increased lipid accumulation and FAS expression, suggesting that HO-1 is upstream of SIRT1 and that suppression of SIRT1 attenuates the beneficial effects of increased levels of HO-1. We also utilized plasmid SIRT to assess if increased expression of SIRT1 (in the absence of HO-1 upregulation) is sufficient to prevent the detrimental effects of AngII on lipid accumulation. Treatment of murine adipocytes with AngII, SnMP, and SIRT plasmid increased lipid accumulation and FAS levels, as compared to murine adipocytes treated with AngII, CoPP, and SIRT1 plasmid (Figure 4A and Figure 4B, respectively). In concordance with our hypothesis, our results further showed that murine adipocytes treated with AngII, CoPP, and SIRT plasmid did not significantly decrease lipid accumulation and FAS levels as compared to cells treated with AngII and CoPP alone, indicating an HO-1-dependent activation of SIRT1 expression. We further demonstrated the mRNA expression of SIRT1, which was significantly reduced by treatment with AngII as compared to the control, was restored by the induction of CoPP (Figure 4C). Concurrent treatment with CoPP and SIRT1-siRNA decreased SIRT1 expression. The utilization of the SIRT plasmid in the group treated with AngII and CoPP significantly upregulated the expression of SIRT1, the effect of which was reversed by treatment with AngII, SnMP, and SIRT plasmid (Figure 4C). 

## 3. Discussion

This study demonstrates for the first time that AngII-induced increased adipocyte dysfunction is accompanied by suppression of cellular SIRT1; effects are reversed by concurrent exposure to CoPP, an inducer of the endogenous antioxidant HO-1. AngII stimulates lipogenesis, oxidative stress, release of inflammatory cytokines, and reduced adiponectin levels in vitro. Our results show the upregulation of MR and increased expression of aldosterone synthase (CYP11B2) by treatment with AngII, an effect that is attenuated by the HO-1-SIRT1 axis. We demonstrated that the alteration in adipocyte phenotype and molecular changes can be reversed in a setting where adipocyte redox balance and SIRT1 is restored by HO-1 upregulation. Hence, our results help establish “the proof-of-principle” of our hypothesis, confirming the beneficial role of the HO-1-SIRT1 axis in adipocytes, further providing a basis that HO-1 can improve adipocyte function by attenuating the activation of AngII expression in adipocytes. 

Oxidative stress is known to be highly involved in the development and progression of clinical conditions like metabolic syndrome. Redox imbalance and chronic oxidative stress increase adipogenesis and cause adipocyte dysfunction [15,31]. We have shown that heme, a pro-oxidant molecule, increases lipid accumulation, promotes cell enlargement, induces over-expression of peroxisome proliferator-activated receptor gamma (PPARɣ), CCAAT enhancer binding protein alpha (C/EBP-α), and adipocyte protein 2 (aP2), and downregulates adiponectin in mouse pre-adipocytes [18,31]. These effects of heme were prevented in cells treated with an antioxidant called tempol, a superoxide dismutase-mimetic. Additionally, in vivo administration of antioxidant reduces visceral adiposity, improves metabolic balance, and restores adipocyte function, as indicated by the recovery of adiponectin levels. Molecular effects of high oxidative stress include suppression of SIRT1, which is amenable to redox manipulations [17]. Our study shows that the upregulation of the antioxidant system by HO-1 induction attenuates AngII-mediated oxidative stress, as shown by the measurement of superoxide levels in our murine pre-adipocytes.

This study highlights the important role of upregulated MR expression in bringing about adipocyte dysfunction. MR is a member of superfamily of nuclear hormone receptors and belongs to the class of ligand-activated transcription factors [32]. Aldosterone and glucocorticoids have similarly high affinity for MR, with Kd values between 0.5 and 3 nM [33]. Inadvertent MR activation in epithelial tissues by circulating glucocorticoids (100- to 1000-fold higher than those of aldosterone) is prevented by the intracellular enzyme 11β-hydroxysteroid dehydrogenase, type 2 (HSD2). HSD2 catalyzes the inactivation of cortisol to cortisone; the latter has negligible affinity for the MR, thus protecting the MR from activation by excess levels of cortisol. Adipose tissues, however, in spite of high MR expression, have minimal HSD2 levels [34]. This sets a stage for aldosterone-mediated increased MR expression in the adipocytes. Congruent studies by other investigators have shown a central role of MR in the lipogenic process. These studies have demonstrated that in an altered pathophysiological condition, increased levels of circulating cortisol diffuse into the adipocytes and bind to MR, further activating it. The activation of ligand-bound MR, which is translocated in the nucleus, stimulates gene transcription, causing an increase in the downstream effectors of MR such as prostaglandin D2 synthase (PTGDS) and genes associated with adipocyte differentiation such as PPARγ and aP2 [35]. In line with these reports, we show that treatment of murine pre-adipocytes with AngII upregulates the expression of CYP11B2, subsequently causing increased expression of MR. Our results also show significant amelioration of these AngII-mediated effects by the induction of the HO-1 antioxidant system through the rescue of SIRT1, which establishes the mechanistic basis of our study.

Evidence has linked upregulated HO-1 expression results in increased insulin sensitivity and improvement in phosphorylation of insulin receptors and adipocyte function [32,33,34,36]. Additionally, induction of HO-1 in adipocyte cell cultures is associated with decreased pro-inflammatory cytokines TNFα and IL-6 [17]. Consistent with these findings, we can see that induction of HO-1 improved insulin sensitivity and decreased levels of TNFα and IL-6 in our murine adipocytes [37]. In concordance with our findings, previously published studies have shown the protective role of HO-1 in inhibiting the inflammatory effect of several mediators. Inflammatory and oxidative transcription factors like nuclear factor kappa-light-chain-enhancer of activated B cells (NF-κβ) and c-Jun N-terminal kinase (JNK) signaling mechanisms, which are primarily involved in inflammatory insult, stimulate inflammatory pathways like IL-signaling, creating a feedback mechanism of inflammation and further compromising pathophysiological conditions [32]. HO-1 have been demonstrated to be effective in suppressing these inflammatory mediators, hence, ameliorating the production of inflammatory cytokines. There is also evidence from the literature that suggests the presence of the HO-1-adiponectin regulatory axis in a murine model [23]. Our results corroborate the findings of the previous studies, as we have shown that HO-1 induction causes an upregulation of adiponectin levels in murine pre-adipocytes. Adiponectin is a protective adipokine, the levels of which are often compromised in a state of excess VAT. A great emphasis has been given to adiponectin recently, due to its role associated with insulin sensitivity and positive effect on triglyceride levels [38,39,40,41]. Reports have also demonstrated that low adiponectin levels are associated with increased oxidative stress [42,43]. Our results show that AngII induces downregulated levels of adiponectin, which contributes toward altered adipocyte phenotype. However, the protective effect of HO-1 is able to increase adiponectin levels, leading to healthier adipocytes. Our study demonstrates that the upregulated HO-1 expression, induced by CoPP, has potential to reprogram the altered adipocyte phenotype to that of a healthy adipocyte by improving oxidative stress, decreasing release of inflammatory cytokines, decreasing lipid accumulation, and increasing adiponectin levels. 

The mechanistic link of AngII exposure observed in our study is provided by SIRT1, which belongs to the family of nicotinamide adenine dinucleotide (NAD)-dependent deacetylases. SIRT1 is a class III protein deacetylase, a crucial cellular survival protein in combating metabolic imbalance [10,44]. SIRT1 is modulated by cellular redox. Resveratrol, an antioxidant, protects SIRT1 against oxidative stress and prolongs longevity in various animal models [45]. AngII activates NADPH oxidases and increases oxidative stress [46,47]. We demonstrate that the oxidative stress induced by AngII leads to attenuation of SIRT1 in adipocytes. SIRT1 rescue and MR-suppression in murine pre-adipocytes treated with CoPP alludes to the protective effect of HO-1 on cellular SIRT1. 

Conclusively, AngII upregulation exerts its effects on oxidative and inflammatory pathways in adipocytes, further inducing phenotypic and molecular changes by inhibiting the HO-1-SIRT1 axis. Our study characterizes that the SIRT1 rescue is HO-1 dependent, which causes reversal of molecular and pathological effects of the AngII cascade in these adipocytes. Our findings are summarized in a schematic representation that demonstrates the AngII-mediated increase in aldosterone synthase, which causes an increase in inflammation, oxidative stress and lipogenesis (Figure 5). This effect is attenuated by the HO-1-induced rescue of SIRT1, hence improving the adipocyte phenotype and molecular changes. This study has far-reaching clinical implications for patients with RAS-dependent metabolic disorders and for patients with secondary RAS activation, systemic or local, as seen in obesity or diabetes. The study elucidates the potential for therapeutic application of HO-1-inducers as a complementary therapy toward abatement of adipose tissue dysfunction, reduction of systemic inflammation, enhancement of adiponectin, and restoration of metabolic balance in these patients.

## 4. Material and Methods

### 4.1. Experimental Design for In Vitro Experiments

Frozen mouse pre-adipocytes (3T3L-1) were purchased from ATTC (ATTC, Manassas, VA, USA). After thawing, 3T3L-1 cells were suspended in Dulbecco’s Modified Eagle Medium (DMEM; Invitrogen, Carlsbad, CA, USA), supplemented with 10% heat-inactivated fetal bovine serum (FBS, Invitrogen, Carlsbad, CA, USA) and 1% antibiotic/antimycotic solution (Invitrogen, Carlsbad, CA, USA). The cells were plated at a density of 1 × 10^6^ cells per 100 cm^2^ dish. The cultures were maintained at 37 °C in a 5% CO_2_ incubator and the medium was changed after 48 h and every ~3–4 days thereafter. Upon attaining confluence, 3T3L-1 cells were recovered by the addition of 0.25% trypsin/EDTA (Invitrogen, Carlsbad, CA, USA). 3T3L-1 cells were plated in 12-well dishes and 75 cm^2^ flasks at a density of 1 × 10^4^. Adipogenesis was initiated at confluence with the adipogenic media (DMEM high glucose with 0.5 mM dexamethasone, 10 µg/mL insulin, and 0.5 mM IBMX). Cells were treated every alternate day with AngII (10 µM), CoPP (5 µM), and SnMP (5 µM) for 7 days in mouse pre-adipocytes. Control groups were treated with adipogenic media alone to induce adipocyte differentiation only, without any treatment with AngII and/or other reagents. We also included an experimental group with our murine pre-adipocytes treated with SnMP alone to demonstrate its inhibitory effects, as previously published [37,48]. 

Commercially available (Ambion Silencer Select) siRNA and an appropriate scrambled RNA for SIRT1 was employed for “knockdown” studies [49]. For overexpression studies, we employed mouse SIRT1, full-length variant (isoform 1, Gene ID93759) synthesized into pJ603 vector, along with corresponding pJ603-GFP negative control by DNA 2.0 Inc. Transfection of cells was achieved using FuGENE HD transfection reagent, as described previously [10].

### 4.2. Oil Red O Staining

Lipid droplets were detected by Oil red O staining. For Oil Red O staining, 0.21% Oil Red O in 100% isopropanol (Sigma-Aldrich, St Louis, MO, USA) was used. Briefly, mouse pre-adipocytes were fixed in 10% formaldehyde, washed in Oil-red O for 10 min, rinsed with 60% isopropanol (Sigma-Aldrich), and the Oil red O was eluted by adding 100% isopropanol for 10 min. The optical density measured at 490 nm, for a 0.5-sec reading. Mouse adipocytes were measured by Oil red O staining (optical density = 490 nm) after day 7 [9].

### 4.3. Western Blot Analysis of IR-β, SIRT1, MR and CYP11B2 

Frozen mouse adipocytes (3T3L-1) were pulverized under liquid nitrogen and placed in a homogenization buffer comprising (mmol/L): 10 phosphate buffer, 250 sucrose, 1 ethylenediaminetetraacetic acid (EDTA), 0.1 phenylmethanesulfonylfluoride, and 0.1% *v*/*v* tergitol, pH 7.5. Homogenates were centrifuged at 27,000 *g* for 10 min at 4°C. The supernatant was isolated and protein levels were assayed (Bradford Method). The supernatant was used for the determination of IR-β, SIRT1, MR, and CYP11B2. Immunoblotting was performed in mouse adipocytes. β-Actin was used to ensure adequate sample loading for all western blots.

### 4.4. Cytokines, Adiponectin, and Lipid Profile Measurements 

Conditioned media (CM) was obtained from our cell culture The levels of interleukin (IL)-6, tumor necrosis factor α (TNFα) and the high molecular weight (HMW) form of adiponectin were determined using an enzyme-linked immunosorbent assay (ELISA) assay kit according to manufacturer’s protocol (Abcam, Cambridge, MA, USA) [50]. Triglyceride levels were measured in CM using an ELISA assay (Assay Gate, Inc., Ijamsville, MD, USA).

### 4.5. Quantitative Real-Time PCR Analysis 

Total RNA was extracted from mouse adipocytes using a 5-Prime PerfectPure RNA Tissue Kit (Fisher Scientific Company, LLC, Waltham, MA, USA). Total RNA was read on a NanoDrop 2000 Spectrophotometer (Thermo Scientific, Wilmington, DE, USA) and cDNA was synthesized using an iScript cDNA Synthesis kit (Bio-Rad, Hercules, CA, USA). PCR amplification of the cDNA was performed by quantitative real-time PCR using a qPCR Core kit for SYBR Green I (Applied Biosystems, Grand Island, NY, USA). The thermocycling protocol consisted of 10 min at 95 °C, 40 cycles of 15 s at 95 °C, 30 s at 60 °C, and finished with a melting curve ranging from 60 to 95 °C to allow distinction of specific products [9]. Primers were designed specific to each gene using Primer Express 3.0 software (Applied Biosystems). Normalization was performed in separate reactions with primers to GAPDH mRNA. Specific primers were used for HO-1 and FAS.

### 4.6. Measurement of Superoxide Levels for In Vitro Experiment 

Mouse adipocytes were cultured on 96-well plates until they achieved approximately 70% confluence. After treatment with or without AngII (10 μM) in the absence and presence of CoPP (5 μM) and SnMP (5 μM) for 2 days, the cells were incubated with 10 μM dihydroethidium (DHE) for 30 min at 37 °C. Fluorescence intensity was measured using a Perkin–Elmer Luminescence Spectrometer at excitation/emission filters of 530/620 nm.

### 4.7. Statistical Analysis 

Statistical significance between experimental groups was determined by the Fisher method of analysis of multiple comparisons (*p* < 0.01). For comparisons among treatment groups, the null hypothesis was tested by a two-factor ANOVA for multiple groups or unpaired t test for two groups. Data are presented as mean ± SE.

## Figures and Tables

**Figure 1:** Effect of Angiotensin II (AngII) exposed to 3T3-L1 murine pre-adipocytes with or without Heme Oxygenase I (HO-1) induction. (**A**) RT-PCR analysis for the relative mRNA expression of HO-1; (**B**) representative images and quantitative data of lipid accumulation measured as the relative absorbance of Oil Red O staining. Images taken with 40× objective lens; (**C**) relative mRNA expression for marker of lipid accumulation, fatty acid synthase (FAS); (**D**) triglyceride levels measured by ELISA assay; RT-PCR analysis for the mRNA expression of (**E**) marker of mitochondrial biogenesis, PGC-1α, and (**F**) inflammatory marker, IL-6. Values represent means ± SEM. * *p* < 0.05 vs. control (CTR), ** *p* < 0.01 vs. CTR, # *p* < 0.05 vs. tin mesoporphyrin (SnMP), ## *p* < 0.01 vs. SnMP, $$ *p* < 0.01 vs. AngII, + *p* < 0.05 vs. AngII + cobalt protoporphyrin (CoPP), ++ *p* < 0.01 vs. AngII + CoPP (*n* = 6).

**Figure 2:** Effect of AngII exposed to 3T3-L1 murine pre-adipocytes by Western blot analysis for protein expression of (**A**) HO-1, (**B**) SIRT1, (**C**) CYP11B2, (**D**) MR, and (**E**) IR-β, shown as mean band densities normalized to β-actin. Values represent means ± SEM. * *p* < 0.05 vs. CTR, ** *p* < 0.01 vs. CTR, ## *p* < 0.01 vs. AngII, ++ *p* < 0.01 vs. AngII + CoPP (*n* = 6).

**Figure 3:** Effect of AngII exposed to 3T3-L1 murine pre-adipocytes on oxidative stress marker, inflammatory marker, and adiponectin levels. (**A**) Superoxide levels assessed with dihydroethidium (DHE) staining; (**B**,**C**) levels of inflammatory markers, IL-6 and TNFα, respectively; (**D**) adiponectin levels. Values represent means ± SEM. ** *p* < 0.01 vs. CTR, # *p* < 0.05 vs. SnMP, ## *p* < 0.01 vs. SnMP, $$ *p* < 0.01 vs. AngII, ++ *p* < 0.01 vs. AngII + CoPP. (*n* = 6).

**Figure 4:** Effect of CoPP with and without SIRT1-siRNA and with and without SIRT plasmid on lipid accumulation and FAS expression in AngII-treated 3T3-L1 murine pre-adipocytes. (**A**) Representative images and quantitative data of lipid accumulation measured as the relative absorbance of Oil Red O staining. Images taken with 40× objective lens; RT-PCR analysis for mRNA expression of (**B**) FAS and (**C**) SIRT1. Values represent means ± SEM. * *p* < 0.05 vs. CTR, ** *p* < 0.01 vs. CTR, # *p* < 0.05 vs. AngII, ## *p* < 0.01 vs. AngII, + *p* < 0.05 vs. AngII + CoPP, ++ *p* < 0.01 vs. AngII+CoPP, $$ *p* < 0.01 vs. AngII + CoPP + SIRT siRNA, & *p* < 0.05 vs. AngII + CoPP + SIRT Plasmid, && *p* < 0.01 vs. AngII + CoPP + SIRT Plasmid (*n* = 6).

**Figure 5:** Schematic representation of AngII-mediated phenotypic alterations in adipocytes, reversed by the HO-1-dependent rescue of SIRT1 in 3T3-L1 murine adipocytes. Each arrow, shown in red, represents the upregulation or downregulation of the respective process.

## Supplementary Materials

Supplementary materials can be found at https://www.mdpi.com/1422-0067/20/13/3205/s1.
